The article "Analysis of the Role of Promoting Sustainable Green Growth through Government Agencies in a Legal Context" was published in 2022. Journal: J Environ Public Health.

# Analysis of the Role of Promoting Sustainable Green Growth through Government Agencies in a Legal Context

**DOI:** 10.1155/2022/6744525

**Published:** 2022-08-25

**Authors:** Hongning Wang

**Affiliations:** School of Law, Jilin University, Changchun 130000, Jilin, China

## Abstract

The rapid development of the global economy has also caused the deterioration of the natural environment. The traditional economic growth method can no longer meet the development requirements of the times for the environment. The realization of sustainable and green development of human society has become the consensus of the whole society. To improve the degree of the greening of the economy, it is necessary to coordinate the management of various departments and to integrate the concept of environment and resources into economic growth. It is an important way for government departments to formulate corresponding sustainable green growth policies by relying on laws to achieve the strategic goals of sustainable green growth. In order to explore the role of government agencies in sustainable green growth through the enactment of relevant laws, this article takes China as the study of the environment. From the perspective of environmental protection tax law, through the establishment of the relationship model between ET and economic variables and ET and environmental indicators, using vector autoregression and system dynamics simulation analysis methods, the effect of ET on the environment and economy is studied. In the analysis of the impact on the environment, the impact of the auxiliary policy of ET on sustainable green growth is discussed. The experimental results show that the impact of environmental tax (ET) on GDP is more obvious. The simulation results show that when the proportion of technology investment is 35%, the promotion effect of sustainable green growth is the best. That is to say, the formulation of relevant laws and policies by government agencies has a certain role in promoting sustainable green growth.

## 1. Introduction

In recent years, with the rapid growth of the global economy, the excessive use of some nonrenewable resources has led to problems such as resource crisis and environmental degradation worldwide. Environmental and resource issues have become challenges that all countries in the world need to face together. The stock of resources on earth is limited. In order to promote economic growth, environmental pollution and ecological damage have been seriously neglected, resulting in massive consumption of energy and resources, and a sharp reduction in nonrenewable resources. Economic losses will be difficult to measure in the future. People are also gradually realizing that if environmental and resource issues are allowed to continue to develop, human beings will pay a high price in terms of economy, personal health, and welfare. All kinds of phenomena show that the traditional growth mode can no longer meet the needs of economic and environmental development in today's society. In this context, human beings need to consider that while maintaining economic growth, resources can continue to provide resources and environmental services to human beings. As a result, a new concept of economic development that can not only meet the needs of economic development but also conform to the concept of environmental protection emerges as the times require, namely, sustainable development strategy and green growth. In order to achieve the strategic goal of sustainable green growth, government agencies need to take effective economic measures. The research on the role and impact of sustainable green growth through a legal perspective can provide theoretical reference for government agencies to establish a sound economic policy for the common development of the environment and economy. It is of great significance to realize the new economic model of sustainable green development.

Starting from the challenges brought about by the environmental and economic problems faced by today's society, this article expresses the necessity of changing the traditional economic growth mode. This leads to the new economic concept of sustainable development strategy and green growth mode. Moreover, from the ET system in the environmental protection tax law implemented by government agencies, the relevant experimental research is carried out on the environment and the economy. According to the search of many literature studies, the research data were obtained from The National Statistical Yearbook of China, and the vector autoregression and system dynamics simulation were used for the study. The results show that the implementation of the environmental tax system has a certain impact on economic growth. Under this premise, legal policies play a supporting role. For example, increasing the proportion of investment in pollution control and technological innovation can effectively achieve the two-way development of economic growth and environmental protection concepts. In short, government agencies have a certain role in promoting the economic development model of sustainable green growth by formulating relevant tax laws. To some extent, this article studies the legal perspective on the research of sustainable green growth, but at the same time, because in the process of data analysis, the environment tax-related data are less, and the concept of environmental taxes is sorted by the literature, there are no official data, it is the limitations of this article, and it is also the direction of further improvement is needed in the future research. The innovation of this article lies in content innovation. At present, there are few studies that integrate the concept of sustainable development and green growth and establish a data analysis model from the perspective of law. Second, the system dynamics simulation is used to analyze the data, the model is tested, and the results are more convincing.

## 2. Literature Review

Protecting the ecological environment while maintaining the economic growth rate is the policy focus of all countries in the world, and many scholars have conducted research on this topic. Podder Bhadra studied the correlation between India's economic growth and the concept of sustainable green development and believed that such a fast-growing economy should pay more attention to the concept of sustainable green development in the process of promoting development [1]. Ali applied the concept of sustainable green development to the green business behavior of banks and analyzed the promotion effect of the sustainable green concept on green banking business through questionnaires [2]. Ge analyzed the sustainable ways to achieve green growth in regions relying on oil economic development by building a system model [3]. Vargas-Hernandez studied the influence factors and contributions of the strategic goals of green economic growth and sustainable development in actual economic transformation through a literature survey [4]. Panzer-Krause analyzed the impact of sustainable green development concepts on the development of rural areas based on a survey of the development concepts of tourism entrepreneurs in rural Ireland [5]. It can be seen that most of these studies on sustainable green growth are aimed at its effects in other aspects, while few of them involve policy research on sustainable green development. An important tool for government agencies to intervene in the market economy is policy, of which taxation is an important part. Therefore, it is necessary to study the ET system constituted by the implementation of economic means.

The ET system is based on the environmental protection tax law. Environmental protection has long been an important issue under the economic development goals of various countries. Sadeleer believed that environmental protection measures should include the formulation of relevant environmental protection tax laws, and analyzed the key issues of levying ET on some large retail enterprises [6]. From the perspective of environmental protection, Yang analyzed the state and pattern of formulating energy use intensity in commercial buildings and investigated the relationship between ET and energy intensity [7]. Zhang carried out a two-layer multiobjective optimization of waste distribution management under the premise of considering ET [8]. Xue Xu analyzed the improvement effect of ET law on urban air pollution through the study of urban air quality [9]. Bassani studied the challenges faced by the ET system between environmental protection and economic compensation [10]. In contrast to existing global-scale studies focusing on semifinished HWP, Zhang has developed a methodology to link global HWP production and end-use by using the Eora multiregional input-output table [11]. Most of these studies are based on the premise of known ET, and research on a single issue of the environment and the economy. Although some of them considered economic issues from the perspective of environmental protection, relatively few of them considered sustainable green development of both environment and economy. However, the environment and the economy are inseparable, and there is a need for coordinated development between economic development and environmental protection. Therefore, it is in line with the needs of the times to explore the influence of relying on the legal system for the coordinated development of economic growth and environmental protection.

### 2.1. Theoretical Deconstruction of Promoting Sustainable Green Growth from the Perspective of Law

#### 2.1.1. Deconstruction of Sustainable Green Growth Theory

Green growth is a circular economy development mode with resource conservation and environmental protection as constraints. Green represents the environment and growth represents the economy, so green growth emphasizes the positive relationship between the environment and the economy [12]. Sustainable development is broadly defined as follows: under the premise of ensuring that natural resources can continue to provide resources and environmental services for the development of human society, it can produce the best results in terms of the economy [13]. It requires people to take into account the resource and environmental needs of future generations while using the natural environment to develop the economy. Green growth is an extended concept of sustainable development theory. At the same time, the strategic goal of sustainable development also provides a leading direction for green growth [14] as shown in Figure 1.

As shown in Figure 1, the basic content of sustainable green growth includes the sustainable development of economy, ecology, and society [15]. Environmental resources on earth are scarce. While pursuing economic development, human beings should also take into account the interests of the next generation and should not blindly pursue economic development. For countries whose industrialization development process is gradually accelerating, the problem of environmental pollution is inevitable. The difficulty is to minimize the problem of environmental pollution. If environmental problems cannot be properly solved, it will also restrict economic growth. Therefore, both developing countries and developed countries need to pay attention to economic development while taking into account the protection of environmental resources, so as to fully realize the goal of green growth [16]. In China, green development mainly includes the content and methods of ecological governance at the micro and macro levels, for example, the integration of green concepts into industrial development to promote industrial upgrading; environmental protection as a part of the green industry has become a new driving force for economic growth and other social phenomena can be called the content of green development. In this process, government agencies need to break through the laws and regulations of ecological governance, integrate the idea of ecological governance into the law, formulate corresponding laws to support ecological governance work, and realize the institutionalization of sustainable green development and the standardization of sustainable green growth [17].

In general, to achieve sustainable green growth, the government, enterprises, and the public need to be united. While achieving economic development and completing the protection of the environment, the state and society should encourage innovation and encourage enterprises and government departments to learn advanced management experience and develop advanced technologies. It is used to seek sustainable green and healthy economic development methods and more efficient organizational models [18], incorporate the concept of sustainable development into the formulation of laws and regulations, and integrate the concept of sustainable green growth into the daily life of the people, so as to better promote its development.

#### 2.1.2. ET System and Its Theoretical Relationship with Sustainable Green Growth

With the increasing problem of environmental pollution, the state has promulgated relevant environmental protection laws and regulations. Among them, the introduction of the Environmental Protection Tax Law is an economic means to reduce environmental pollution while maintaining economic growth under the market economy. The ET under the Environmental Protection Tax Law mainly refers to some taxes with green properties. The theoretical relationship between ET and sustainable green growth is shown in Figure 2.

As shown in Figure 2, the content of sustainable green growth includes three aspects: economy, environment, and society. A complete sustainable green growth system is the balanced development of these three aspects. Energy resources in the environment can bring value to the economy, and while realizing economic value, attention should be paid to maintaining environmental quality and having a good natural environment and economic level. Humans will have more social welfare, which is an interlocking cyclic process. In order to realize this whole process perfectly, enterprises, institutions, and individuals need to have good environmental awareness. Government agencies should encourage society to realize technological innovation and formulate relevant laws and policies for pollution control [19]. Appropriate subsidies should be given to encourage enterprises to move closer to the concept of sustainable green growth while collecting environmental taxes.

From the relationship between the two, the ET system can promote sustainable green development. This is because the effective implementation of the ET system can solve the problems of unreasonable resource allocation and environmental pollution control to a certain extent. A good and harmonious resource and environment is an important prerequisite for achieving sustainable green growth. From another perspective, the implementation of the ET system and the legalization of the concept of protecting the ecological environment for people from all walks of life are conducive to promoting the process of sustainable green development in the whole society. Therefore, it can be said that ET can actually provide the necessary guarantee for sustainable green growth. These tax revenues can provide corresponding financial support for environmental pollution control [20]. In this process, the environmental cost of enterprises has increased, which can effectively restrain the current situation of excessive environmental development and pollution and effectively achieve the purpose of environmental protection. In recent years, the government has reduced the frequency of consumers' use of products that can cause environmental damage through price regulation, which is also a manifestation of sustainable green growth. For example, the rise in gasoline prices has promoted the increase in sales of new energy-saving vehicles, indicating that the implementation of the ET system can promote the sustainable development of people's consumption behavior [21, 22]. All in all, from a theoretical analysis point of view, the environmental tax system can effectively promote sustainable green growth.

#### 2.1.3. Sustainable Green Growth Evaluation

In recent years, the theory of sustainable green growth is developing constantly. The concept of green growth is not only limited to theory, but also gradually begins to develop into practice. Therefore, how to judge the fit degree of green growth theory and practice, that is, how to evaluate the actual results of green growth in practice, is an important step for green growth to be successfully practiced from theory. Therefore, it is necessary to objectively evaluate the contribution of green growth to reality. At present, the evaluation index system mainly focuses on the evaluation system established by international authoritative institutions, experts, and scholars around the world. Among them, international authorities include OECD, UNEP, WB, and GGGI. The rating indicators established by OECD are evaluated from these aspects: economic background and growth characteristics, environmental resource productivity, natural resource base, environmental quality, economic development opportunities and policy support, and correlation with green growth, rationality analysis, and data scalability. UNEP constructs evaluation indicators from three aspects: environmental problems and development goals, green economic measures intervention, and the relationship between green economic measures and society. WB takes society, economy, and environment as the overall framework and constructs from the aspects of environmental quality improvement, consumption of human material resources and natural resources, employment, and so on. GGGI takes the country as the basic consideration unit and designs the evaluation index comprehensively from the perspective of the country's general situation, development, and support. The evaluation indicators established by experts and scholars around the world are basically based on international authoritative institutions and modified according to the characteristics of the study area. This article will integrate the evaluation indicators of international authoritative institutions and study sustainable green growth from the aspects of environment and economy.

### 2.2. Deconstruction of the Role of Promoting Sustainable Green Growth from a Legal Perspective

#### 2.2.1. Data and Variables

This article conducts relevant research on the cycle system of sustainable green growth, and defines variables from the aspects of economy, environment, society, and ET. First, economic variables include GDP, urban unemployment rate, and consumer price index (CPI); environmental variables include wastewater, waste and solid waste (three wastes) emissions, energy consumption, and pollution index [23]. Social variables include the Human Sustainability Index (HSDI) adjusted for unevenness. ET supporting policies are reflected in pollution control, technology investment, and general user subsidies. This article will study the impact of these supporting policies on the environment.

The pollution index mainly measures the impact of the “three wastes” on the environment, and its calculation formula is as follows:

(1) $$\begin{array}{c} \lambda_{a}=\sum_{b=1}\omega_{b}\delta_{ab}. \end{array}$$

Among them, a represents the year, *b* represents the number of pollution indicators, *δ* represents the proportion, and *ω* represents the weight.

The HSDI is composed of health, education, income, and pollution index, and its calculation formula is as follows:

(2) $$\begin{array}{c} HSDI=\sum_{T=1}^{R}\frac{{\left(M_{T}-N_{T}\right)}^{Ginl}}{\left(K_{T}-M_{T}\right)R}. \end{array}$$

According to the data from China's National Statistical Yearbook, the environmental protection tax revenue has had specific values since 2018. The data for the past three years are shown in Table 1.

As shown in Table 1, the environmental protection tax in the past three years has not accounted for a small proportion of the total tax revenue, and the data are relatively small. Therefore, this article will select other tax revenue related to environmental protection for relevant analysis, which can explore the impact of environment-related tax regimes on the economy and the environment. All these environment-related taxes are collectively referred to as ET, and the details are as follows. For example, value-added tax, consumption tax, and enterprise income tax reflect economic aspects; in terms of land, urban land use tax and farmland occupation tax; it also includes resource tax and vehicle purchase tax. According to the data from China's National Statistical Yearbook, the ET revenue data from 2011 to 2020 are shown in Table 2.

As shown in Table 2, in general, the ET revenue generally increases year by year, with a few taxes increasing and decreasing. In order to better reflect the greening degree of taxation, the total ET revenue and total tax revenue and their ratios are drawn into a statistical figure, as shown in Figure 3.

As shown in Figure 3, during the period from 2011 to 2020, ET revenue increased almost year by year. In 2020, affected by the pandemic, various tax revenues decreased. The proportion of ET revenue grew the fastest between 2015 and 2017 and was relatively stable after that, which also shows that the implementation of ET needs to be improved.

The data of GDP, urban unemployment rate, and consumer price index from 2011 to 2020 are shown in Table 3.

The emissions and total energy consumption of the “three wastes” from 2011 to 2017 are shown in Table 4.

The data in Tables 3 and 4 are all from the National Statistical Yearbook of China. This article will use these data to explore the impact of environmental taxes on the economy and the environment.

### 2.3. Deconstructing the Role of ET on the Economy

First, according to the data contained in Figure 3 and Table 3, it is assumed that ET is conducive to sustainable economic growth. Next, the vector autoregressive model will be used to test the hypothesis, and the impulse function will be used to analyze the vector autoregressive model. The obtained experimental results are shown in Figure 4.

As shown in Figure 4, when the ET is given a positive shock, the responses of GDP, urban unemployment rate, and CPI are observed, respectively. From the perspective of GDP indicators, GDP rose gradually in the early stage, but the increase was not large. Then, there was a negative growth in GDP, indicating that the ET had an inhibitory effect on GDP. However followed by growth again and again, the magnitude of the role was getting bigger and bigger, indicating that the impact of ET on GDP is more notable. Judging from the urban unemployment rate indicator, in the initial stage, the curve is downward; it can be seen that the ET has a restraining effect on the unemployment rate, but there is almost no change after that. It shows that the ET has an impact on employment promotion only at the beginning, but in the long run, this impact is negligible. The same is true for CPI. The trend of change is similar to that of the unemployment rate, and there is almost no change in the later period. It shows that the impact of ET on CPI is very weak, that is to say, prices will not fluctuate greatly because of ET.

According to the analysis of the above three functions, it can be concluded that the impact of the ET system on GDP is relatively obvious. This effect circulates between inhibition and promotion, and the force gradually increases. This shows that government agencies implement an effective ET system, which has a greater impact on the economic aggregate. Overall, the ET system can effectively promote the realization of sustainable green growth. However, in terms of employment and prices, the impact of ET is minimal, indicating that the implementation of the ET system does not affect people's employment and consumption levels. From this, it can be shown that environmental taxes mainly have an impact on GDP in economic variables.

### 2.4. Deconstruction of the Effect of ET on the Environment

The analysis of the environment will be carried out with two variables, pollution index and HSDI. Predictive analysis of these two indicators is carried out through system dynamics simulation. First, the validity of the model is verified. This article will test the consistency between the retrograde simulated value and the real value, and the test results are shown in Figure 5.

It can be seen from the data in Figure 5 that the average absolute error between the simulated value and real value of GDP and the total energy consumption is 4.85% and 4.98%, respectively, and the simulated value is basically consistent with the real value, indicating that the variable selection and parameter setting of the model and the functional relationship between variables are reasonable.

During the experiment, in order to better observe the impact of ET and its supporting policies on the environment, three groups of schemes were designed for comparison. Among them, group A represents the situation where there is no investment in ET and its related content, as a control group, group B represents the participation in ET but no investment in other related policies, group C is in the case of adding ET, and the investment in other related policies is the same. The proportion of investment is 20%. The obtained simulation results are shown in Figure 6.

As shown in Figure 6, when the ET is added and there is no support for other related policies, the pollution index decreases. It shows that the emission of pollutants has been alleviated, but the mitigation extent is not large. When the ET was added and the relevant policies were invested, the pollution index decreased significantly. It shows that while levying ET, encouraging enterprises to carry out technological innovation and providing subsidy support has a certain effect on curbing environmental pollution. The simulation results of HSDI also show that when the ET is levied alone and supplementary support is added, the HSDI has a certain increase, but the increase is small. After adding auxiliary support, the increase is larger. However, in the long run, the change in HSDI shows a downward trend. It shows that after adding ET and its auxiliary policies, the environment can be improved within a certain period of time, but the environmental cost will also increase, which will bring pressure on the economy and society. In general, the collection of ET and supplementary policy support can achieve a better effect on sustainable green growth.

From the simulation results, the simultaneous implementation of ET and related policies is more conducive to the sustainable development of the environment and economy. Next, it will be discussed how to adjust the investment ratio of auxiliary policies under the premise of adding ET. That is, pollution control, technology investment, and general user subsidy investment are simulated and analyzed according to different investment ratios. Under the premise that the environmental tax conditions remain unchanged, the input ratios of the three control groups are set to be 20%, and the experimental groups are groups D, E, and F. Based on the control group, the investment ratios for the three policies were increased by 15%. The proportion setting of each group is shown in Table 5.

As shown in Table 5, the setting ratio of the simulation was carried out according to the content of Table 5, and the obtained simulation results are shown in Figure 7.

As shown in Figure 7, when the input ratios of the three auxiliary policies are inconsistent, the effects on the pollution index and HSDI are also inconsistent. It can be seen that when the technology investment ratio is the highest, the environmental pollution index is the lowest, and the HSDI value is the highest. It shows that increasing the support for technology has a greater effect on promoting sustainable green growth, and the proportion of investment in increasing pollution control is slightly better than that in user subsidies. On the whole, under the conditions of the implementation of ET, appropriate investment in technology should be given, and the proportion of funds for pollution control should be increased accordingly, which will play a better role in the development of the green economy.

From the above two sections, it can be seen that environmental tax has a certain impact on environmental protection and economic growth. Moreover, its effect on GDP is more obvious, its effect is cyclical, and its effect on GDP increases year by year. In terms of employment and prices, environmental tax has little impact on these two aspects, indicating that the economic and employment dividend brought by the environmental tax is not significant at present. From an environmental point of view, increasing investment in technology is more conducive to sustainable green growth.

## 3. Conclusion

This article explores the relationship and retrograde between ET and sustainable green growth by constructing an analytical model. Comprehensive economic and environmental analysis shows that ET has a more obvious role in promoting sustainable green growth. In terms of the economy, adding ET has an obvious effect on economic growth, but has little effect on the unemployment rate and consumption level. In terms of the environment, adding an ET can effectively reduce the emission of pollutants and increase the level of HSDI. Under the condition of ET, supplemented by supporting policies, such as technology investment and pollution control investment, the improvement effect on the environment is the best. In general, it can be concluded from the related research in this article: first, the ET can be increased in the initial stage, but it should be appropriately reduced in the long run. This is due to the large amount of pollutants discharged in the initial stage. At this time, increasing the ET can achieve a good restraint on such behaviors of enterprises. With the passage of time, the emission of pollutants is less, and the improvement effect will be significantly weakened by continuing to implement the original policy at this time. Second, auxiliary policies should be properly equipped with the collection of environmental theory, especially the technical innovation of enterprises can be given corresponding support. To a certain extent, this can better achieve the goal of sustainable green growth. In general, government agencies have a good role in promoting sustainable green growth by formulating relevant laws and policies and supplemented by supporting policies. The concept of sustainable green growth has been put forward so far. Relevant research on action path, evaluation index, and other aspects is mainly based on the macro level, but the research on the micro level of a certain industry or enterprise needs to be further pursued. At the same time, according to China's official data, from the legal angle, using the authority of a government that has set up the environment tax that is collected and measures that are still in their infancy, it is only appropriate to change, on the basis of blowdown cost in the future, how legal means are used to promote sustainable green growth, which is the focus of subsequent research.

## Figures and Tables

**Figure 1:** Basic elements of sustainable green growth.

**Figure 2:** Theoretical relationship between ET and sustainable green growth.

**Figure 3:** ET and their proportions.

**Figure 4:** Response functions between ET and several economic variables. (a) Response curve of GDP to ET. (b) Response curve of urban unemployment rate to ET. (c) Response curve of consumer price index to ET.

**Figure 5:** Fitting diagram of simulated value and real value. (a) Fitting graph of simulated GDP and real GDP. (b) Fitting diagram of simulated value and real value of total energy consumption.

**Figure 6:** Pollution index and HSDI simulation results under different scenarios. (a) Simulation results of a pollution index. (b) HSDI simulation results.

**Figure 7:** Pollution index and HSDI simulation results under the adjustment scheme. (a) Simulation results of the pollution index. (b) HSDI simulation results.

**Table 1:** 2018–2020 environmental protection tax data.

Year	Environmental protection tax revenue (100 million yuan)	Total tax revenue (100 million yuan)	Proportion (%)
2018	151.38	156402.86	0.097
2019	221.16	158000.46	0.140
2020	207.06	154312.29	0.134

**Table 2:** ET revenue data from 2011 to 2020 (100 million yuan).

Year	Added value tax	Consumption tax	Corporate income tax	Resource tax	Urban maintenance and construction tax	Urban land use tax	Vehicle purchase tax	Farmland occupation tax
2011	24266.63	6936.21	16769.64	595.87	2779.29	1222.26	2044.89	1075.46
2012	26415.51	7875.58	19654.53	904.37	3125.63	1541.72	2228.91	1620.71
2013	28810.13	8231.32	22427.2	1005.65	3419.90	1718.77	2596.34	1808.23
2014	30855.36	8907.12	24642.19	1083.82	3644.64	1992.62	2885.11	2059.05
2015	31109.47	10542.16	27133.87	1034.94	3886.32	2142.04	2792.5916	2097.21
2016	40712.08	10217.23	28851.36	950.83	4033.60	2255.74	2674.16	2028.89
2017	56378.18	10225.09	32117.29	1353.32	4362.15	2360.55	3280.67	1651.89
2018	61530.77	10631.75	35323.71	1629.90	4839.98	2387.60	3452.53	1318.85
2019	62347.36	12564.44	37303.77	1821.64	4820.57	2195.41	3498.26	1389.84
2020	56791.24	12028.10	36425.81	1754.76	4607.58	2058.22	3530.88	1257.57

**Table 3:** Data on some economic variables from 2015 to 2017.

Year	GDP (100 million yuan)	Urban unemployment rate	Consumer price index (CPI)
2011	487940.2	4.1	109.8
2012	538580.0	4.1	109.1
2013	592963.2	4.05	107.9
2014	643563.1	4.09	108.4
2015	688858.2	4.05	109.5
2016	746395.1	4.02	108.2
2017	832035.9	3.9	106.6
2018	919281.1	4.9	107.4
2019	986515.2	5.2	106.1
2020	1015986.2	5.2	97.8

**Table 4:** Emissions and total energy consumption of “three wastes” from 2011 to 2017.

Year	Wastewater discharge/ten thousand tons	Exhaust emissions/ten thousand tons	Solid waste output/ten thousand tons	Total energy consumption (tons of standard coal)
2011	6591922	5901.01	322772.34	387043
2012	6847612	5691.16	329044.26	401238
2013	6954433	5549.42	327701.94	416913
2014	7161751	5793.17	325620.02	428334
2015	7353227	5248.15	327079	434113
2016	7110954	3507.83	309210	441492
2017	6996610	2930.49	331592	455827

**Table 5:** Group ratio settings.

Group	Proportion of investment in pollution control (%)	Proportion of technology investment (%)	Proportion of subsidy input for general users (%)
Control group	20	20	20
D	35	20	20
E	20	35	20
F	20	20	35

## Data Availability

The data used to support the findings of this study are available from the corresponding author upon request.
